# Load Balancing Algorithms for Hadoop Cluster in Unbalanced Environment

**DOI:** 10.1155/2022/1545024

**Published:** 2022-10-07

**Authors:** Weiyu Fu, Lixia Wang

**Affiliations:** ^1^School of Computer Science and Technology, China University of Mining and Technology, Xuzhou, Jiangsu 221116, China; ^2^Jiangsu Vocational College of Finance and Economics, Huai'an, Jiangsu 223003, China; ^3^School of Management, China University of Mining and Technology, Xuzhou, Jiangsu 221116, China; ^4^School of Business Administration, Henan Polytechnic University, Jiaozuo, Henan 454003, China

## Abstract

Considering that in the process of job scheduling, the cluster load should be prebalanced rather than remedied when the load is seriously unbalanced; therefore, in this paper, the task scheduling flow of the Hadoop cluster is analyzed deeply. On the Hadoop platform, a self-dividing algorithm is proposed for load balancing. An intelligent optimization algorithm is used to solve load balance. A dynamic feedback load balancing scheduling method is proposed from the point of view of task scheduling. In order to solve the shortcoming of the fair scheduling algorithm, this paper proposes two ways to improve the resource utilization and overall performance of Hadoop. When the mapping task is completed and the tasks to be reduced are assigned, the task assignment is based on the performance of the nodes to be reduced. It gives full play to the advantages of the ant colony algorithm and the hive colony algorithm so that the fusion algorithm can better deal with load balance. Then, three existing scheduling algorithms are introduced in detail: single queue scheduling, capacity scheduling, and fair scheduling. On this basis, an improved task scheduling strategy based on genetic algorithm is proposed to allocate and execute application tasks to reduce task completion time. The experiment verifies the effectiveness of the algorithm. The LBNP algorithm greatly improves the efficiency of reducing task execution and job execution. The delay capacity scheduling algorithm can ensure that most tasks can achieve localization scheduling, improve resource utilization, improve load balance, and speed up job completion time.

## 1. Introduction

With the popularity of the Internet and the growing maturity and perfection of related technologies, the impact of the Internet on our work, learning, and life is growing. It improves our work and study efficiency, changes our study and life style, and improves our quality of life [1]. At the critical moment of processing massive data, cloud computing technology comes into being. So far, many network companies have their own cloud computing systems at home and abroad, and they invest a lot of money every year as the main direction of future development [2]. At present, many Internet companies are mining valueable information from a large number of user data and predicting the potential behavior of users, resulting in a certain commercial value. Future storage modes will change the current storage mode, no longer stored on personal computers and servers but stored on cloud servers. At the same time, all computing and processing work will be completed on cloud servers. In Hadoop clusters, the performance consumption of mobile data blocks is higher than the performance consumption of mobile computing tasks, and data load balancing can improve the number of localized tasks [3]. In this project, not only IT expertise but also related domain knowledge is required. At the same time, various software and hardware infrastructures are needed. In addition, the processing of big data requires more and more storage space and computing resources, and the overhead of traditional processing methods is also increasing [4]. Therefore, facing big data processing technology has become a new challenge.

The era of big data is a special era. It will open up the challenge of massive data to traditional technologies. The analysis and processing of massive data in the era of big data has many different places for data analysis and processing. For example, it is no longer just concerned with samples but focuses on the whole [5]. Hadoop is a secure, reliable, and parallelizable open source framework that implements transparent processing for application developers without the need to understand the underlying implementation details of Hadoop. As people pay more attention to data, data have penetrated into every aspect of political and economic activities. As people pay more attention to big data, its application is also expanding [6]. Hadoop has unparalleled advantages in many cloud computing products, and more and more Internet companies' massive data solutions are preferred to use the Hadoop open source project. The traditional way of processing is to use a processor as the center, and then to process data through data movement [7]. In the environment of large data, the huge amount of data will bring great inconvenience to data movement. It is no longer just looking for causality, but more looking for correlation to find more meaningful value between data hidden behind massive data [8]. Job scheduling technology is the core technology of the Hadoop platform. It is mainly responsible for allocating idle resources to each job in the system and controlling the sequence of job execution. It plays a vital role in computing resource allocation and the overall performance of the Hadoop platform.

In Hadoop, users can not only use the data in the default format of the system but also store and analyze the data in a customized format, so they can store and analyze all kinds of data [9]. This paper analyses the shortcomings of setting delay time interval in delay scheduling algorithm, clarifies the importance of delay time interval to localized scheduling, and gives a reasonable setting scheme of delay time on the basis of retaining the conciseness and efficiency of the delay scheduling algorithm, so as to make the delay scheduling algorithm play its optimal efficiency [10]. When small jobs are submitted late, the actual execution time may be much less than the waiting time, and if there are several large jobs that need to be run for a long time before, the waiting time will be more. Therefore, we have important significance for the study of job scheduling algorithms. The task scheduling algorithm is considered a complex process because it must make full use of the available resources to perform a large number of tasks [11]. It simplifies the file consistency model when it is stored. It can streamline the throughput of data access and adapt to applications with large data sets. This paper describes the data load balancing algorithm of Hadoop first described and then proposes an improved load balancing algorithm through a large number of experiments. It is proved that the improved algorithm can balance the data load of each rack in a specific time.

In this paper, we propose a research model of the Hadoop cluster load balancing algorithm based on an unbalanced environment, which is an analysis model of the Hadoop cluster load balancing algorithm. In summary, our contributions are as follows:

1. This algorithm is an analysis model based on an unbalanced environment for the research of load balancing algorithm in the fast Hadoop cluster.
2. This paper proposes an analysis model for Hadoop cluster load balancing algorithm research.
3. This model is widely applicable to the analysis of load balancing algorithm for Hadoop cluster, and it has higher efficiency, wider applicability, and higher recognition.

## 2. Related Work

What strategies should be adopted to balance the overall load of the cluster and improve the utilization of resources in the cluster has become a research hotspot for scholars at home and abroad. Equitable allocation of task resources is a key factor in the Hadoop cluster. It mainly guarantees not only the efficiency of job execution but also the fairness among users under multiuser task operation [12]. Qureshi et al. propose a fair scheduling algorithm, which uses resource pools to run jobs [13]. Javanmardi et al. pointed out that considering fairness cannot take efficiency into account, and considering efficiency cannot take good care of the fair distribution of resource slots, so the author tried to consider these two factors at the same time and allocate resources fairly and reasonably to submitted jobs [14]. Lim et al. studied the load problem of Reduce [15]. Strutz et al. use an object-based cluster sampling method when evaluating Reduce loads. The overloaded key is divided into subkeys and the subkeys are assigned to reduce implementation [16]. Zhou et al. proposed an enhanced task scheduling algorithm based on GA. They mainly made changes to the fitness function, using a new fitness function based on the average [17]. However, since the static algorithm does not consider the current load of each machine in the cluster, it is not very good for load balancing.

Zhang et al. proposed a computing resource allocation algorithm based on ant colony optimization, which uses the optimization algorithm to obtain an optimal resource allocation scheme and improve resource utilization [18]. The fair scheduling algorithm can ensure that each user submitting the job gets a response within a certain period of time, which is very fair. On the basis of the fair scheduling algorithm, Singh and Kaur proposed an improvement based on the Hadoop fair scheduling algorithm, which satisfies the priority job processing as much as possible while ensuring fairness, and considers the operation of low-priority jobs [19]. The scheduling algorithm proposed by Yao et al. can schedule jobs according to the weights of jobs, but the weights of jobs can be directly interacted with the system by the tools provided by the system. It can dynamically change the weights of jobs when the program runs, so as to directly interfere with the scheduler [20]. Ibrahim et al. studied the randomness of HDFS copy selection and proposed a new backup node selection strategy. This strategy considers the disk usage of nodes when selecting nodes for backup data blocks [21]. In the cloud computing platform based on the Hadoop framework, the computing resources and the required data resources may be located in different physical locations. When the data required by the computing resources are in different locations, the data needs to be migrated. This is the so-called data localization problem. Only when the data and the computing task are in the same node can the computing efficiency be guaranteed [22, 23]. Therefore, the degree of data localization is an important factor that determines the efficiency of cloud computing under the Hadoop framework. These tasks are sorted, and then the first task in the queue is acquired and allocated to the most suitable resource obtained by GA to complete the scheduling. The goal of this strategy is to maximize the use of resources while reducing execution time.

## 3. Methodology

The Hadoop ecosystem refers to the Hadoop platform with multiple subprojects. Early Hadoop consisted of three subprojects: Hadoop Common, HDFS, and Hadoop Map Reduce. It enables transparent processing of application developers [24, 25]. Users can easily use Hadoop to integrate computer resources to build their own computing platform and complete massive data processing without knowing the details of Hadoop's underlying implementation. Hadoop provides users with a basic distributed architecture on which developers can directly develop highly scalable distributed applications. And they can focus only on the logic of the application, without paying attention to the details of the distribution [26]. Because the disk space of each node is different in a heterogeneous cluster environment, the theoretical amount of space used for each node calculated may be greater than the maximum load of the node. Each private cluster has independent schedulers and uses its own scheduling algorithm to manipulate its own resources, reducing the competitive requirements of the operations on resources [27]. In addition, the jobs run independently in their own clusters, and jobs from different users can be executed simultaneously. Hadoop's business is usually composed of a single-user large-scale batch task, which is sent to a unique job queue in the order in which the jobs are submitted, and the job priority is determined by [28, 29].

The Hadoop Map Reduce model consists of the following phases: setup, mapping, out-of-order processing, sorting, and reduction, as shown in Figure 1. The Hadoop framework consists of a master node and a cluster of compute nodes. Jobs submitted to Hadoop will be further distributed to the map and reduced tasks [30]. In the setup phase, the input data of the job to be processed are logically partitioned into the same volume, which is called the block mapping the working node. Hadoop divides each Map Reduce job into a set of tasks, each of which is handled by a map worker.

The user who uses the cluster really cares about the response time of the job. Therefore, in this different scheduling mode, Word Count executes one job ten times and calculates the average response time of the job. The average response time for executing Word Count 10 times is shown in Figure 2.

Hadoop Map Reduce draws heavily on the design of Google Map Reduce in terms of simplifying programming interfaces and improving system fault tolerance. This idea is generated in the field of search, and its role is to deal with the problem of insufficient scalability in the calculation of massive data that is prevalent in search engines at the time. Running on Hadoop, it provides a platform for large-scale data analysis and evaluation, a high-level programming language that reduces the need to use Hadoop [31]. The Hadoop distributed file system (HDFS) is used as the master node to manage and distribute the massive data input. The upper layer distributed data processing (Map Reduce) processes the distributed data and finally outputs it. This structure greatly improves the processing efficiency of the whole system. Hadoop's core framework provides basic services for building large-scale distributed architecture on low-cost commercial hardware, as well as interfaces for running software in this system [32]. The number of bytes that can be balanced between two pairs of nodes equalizes as many bytes as possible. For the source node, if the number of bytes that have been balanced after balancing is greater than the number of bytes that need to be balanced, the balance is considered to be over. Then the theoretical space usage is calculated by the percentage of the performance of each node to the total performance, and then the theoretical space usage rate is calculated. No matter the size of the two jobs or the order of arrival, because they belong to different users and have their own scheduling resources, they are independent of each other, without the influence of competitive resources, and can be executed independently at the same time.

Figure 3 below describes the architecture of the REST-Map Reduce framework. It has five core components. First, the REST-Map Reduce request processor acts as a service differentiator in this framework. It determines whether the incoming request is REST, Open API, or Map Reduce. It is then sent to Hadoop according to the type of request.

Jersey provides an API so developers can extend Jersey to meet their needs. We use Tomcat and Jersey to implement our system. We built an eight-node Linux core i5 machine cluster with 4 gigabytes of RAM per cluster. These machines are connected through the network and managed by Hadoop.  Figure 4 shows an overview of our REST Map Reduce framework architecture.

The fair scheduling method supports job pre-emption. When a new job appears in the system, the new job will wait for the work node to complete the previous task, then release the task slot and assign it to the new job. Usually, in order to improve the overall performance of the cluster, an effective and reasonable load balancing algorithm should be used to make the amount of data allocated to each node basically the same. Storage of loose data can provide real-time and random access to large data. In addition to row and column keys, keys also add time stamps, and data columns can be dynamically increased. Its reliability, fault tolerance, expansibility, and high efficiency bring great convenience to the data storage of the Hadoop platform. At the same time, it also provides the function of management and assignment of tasks and submits jobs to Map Reduce. All input data is first parsed into a bar key value pair, and then processed by a user-defined function. After the process is completed, the data is handed over to the user-defined Reduce function through the Shuffle phase. Calculate the maximum spatial load rate of each node, and thus find the node whose theoretical space usage exceeds the maximum load, calculate the excess, and place the excess space as the excess node. The jobs of different users are different. The size of the jobs submitted to the specific private group is different from the number of jobs. Therefore, the load between the private groups must be very different. The most obvious difference is a private one. Groups are idle, and a private group is overloaded.

## 4. Result Analysis and Discussion

Hadoop tasks are classified as data-intensive, computationally intensive, etc., depending on the type of job. For heterogeneous, data-intensive computing environments, one of the cores of data-intensive computing is to replace mobile data with mobile computing as much as possible. Poor scheduling in a Hadoop cluster can result in uneven load on the cluster, resulting in high overall cluster load and long processing time. The balanced load tool in Hadoop balancer is only used when the Data Node disk usage is too high you must manually start the program to adjust the node disk file. During Hadoop's execution of tasks, it is sometimes necessary to connect multiple Map/Reduce jobs together to accomplish larger tasks, and there may be dependencies between these jobs. The Hadoop distributed file system (HDFS) is a kind of cost-saving distributed file system, which is usually deployed on cheap hardware. Its design purpose is to be a commercially distributed file system. Compared with the existing distributed file system, it has many similarities and many differences. It draws lessons from the design concept of the former. The HDFS is responsible for data storage management. It can run on low-cost computers and achieve fault-tolerant performance of the system by detecting and responding to hardware failures. It has been distributed on the data nodes. In the HDFS source code of Hadoop, a random algorithm is used to select data nodes to store data. Therefore, during the initialization of the simulation experiment, the data node is also directly selected randomly as the physical storage location of the data slice. The main part of the scheduling algorithm remains the original. The initialization simulation system is a cluster of 1000 and 2000 nodes, and each node is equipped with a resource slot. Submit jobs with different lengths when the expected localization probability is 70%, 80%, and 90%. Experiments show that for the total balance time, sometimes the algorithm takes a shorter time and sometimes the improved algorithm takes a shorter time, which is related to the different strategies of data computing and moving. Therefore, the input data must be copied remotely before running the task.

The Map function takes a log line, takes out the time stamp field when the server completes processing the request, converts it into a slot of one minute a week, and writes it to the file system. Reduce phase reads and sorts all intermediate data to combine all occurrences of the same key to get the final result of digitally adding all the same keys, as shown in Figure 5.

Let the number of partitions of the Map result be l, the number of nodes be *t*, and the amount of data of the *y* partition on node *t* be denoted as *S*. Then the execution time of all partitions on node *t* is expressed as:

(1) $$\begin{array}{c} S\left(t\right)=\frac{y\left(t\right)}{l}\text{.} \end{array}$$

If the total amount of data on node *j* after partition allocation is *R*, then the maximum time difference of the total processing time of cluster tasks is estimated by the following formula:

(2) $$\begin{array}{c} k_{j}=\frac{R_{j}}{Dj}\times Uj\times {\text{Re}}_{j}\text{.} \end{array}$$

Taboo table *f* is set to record the list of cities that ant *I* has completed traversing. *R* is used to express the probability of ant *J* transferring from *I* city to *J* city at time *T*. The formula is as follows:

(3) $$\begin{array}{c} R_{j}=\frac{f_{ij}}{Tj}\times S_{j}\text{.} \end{array}$$

*S* represents a pheromone residual factor. After all ants have cycled in each city for a week, the pheromone concentration on each road between cities is updated as follows:

(4) $$\begin{array}{c} S_{j}=\frac{1}{\sum_{i=1}^{n}\left(S_{r}\right)},\left(0<\left(S_{j}\right)\leq 1\right)\text{.} \end{array}$$

The selection operation is that individuals with high fitness calculated by fitness function are inherited according to certain rules, and the higher the fitness, the greater the probability of being selected. Here, we use fitness probability to determine the probability of individual selection, and the probability to determine the number of individuals selected.  Figure 6 shows individual fitness probability and a selected random number.

The algorithm can obtain the quantitative index of the node's performance, and the cluster data is placed according to the node's performance ratio, so that the machine with good performance places more task data and the performance node is preferentially selected when performing data backup. The pros and cons of the scheduling algorithm will directly affect the execution efficiency of the jobs in the cluster, and the efficient scheduling algorithm will bring great convenience to the job processing. In the processing of large-scale data, the entire calculation process is not terminated due to errors in some nodes in the Hadoop cluster. In addition, the HDFS has a relatively complete redundant backup and fault recovery mechanism, enabling reliable mass file storage. Since ordinary cheap machines are prone to failure, HDFS is designed to take hardware failures as a normal state and can quickly detect and eliminate faults in the event of a fault. It can store some unstructured and semistructured data. It is Google Open source implementation of the file system Big Table, which can provide scalable and high-performance dynamic data services for various types of data. In HOD, because the scheduler in the private cluster is in charge of its own computing resources, tasks submitted to a private cluster are only scheduled to run in the nodes of the private cluster, which reduces the scope of resources available to jobs. The resource utilization of the whole system is not satisfactory. In addition, because the next job must wait for the completion of the previous job before it can be selected to be executed, this algorithm is very disadvantageous for the processing of small jobs.

To evaluate the effectiveness of the whole HDFS data placement strategy improvement algorithm, two aspects should be considered: the load balance of the cluster and the efficiency of the cluster. To judge whether the cluster is balanced or not, we judge the efficiency of the cluster by judging the load of the node for a period of time. We use the job execution time of Map Reduce to judge.  Figure 7 shows node load assessments.

The optimization target selected by the algorithm is the load deviation degree, and the standard deviation calculation method is used, that is, the standard deviation *D* of the load of each node of the cluster is used to represent the cluster load, and the formula is as follows:

(5) $$\begin{array}{c} D_{j}=\overset{n}{\underset{i=1}{\sum }}\left(H_{P}\times V_{p}\right)\text{.} \end{array}$$

*S* denotes memory usage of node *i*, *r* denotes bandwidth usage of node *i*, *w* denotes disk usage of node *i*, hence the load factor of node *i* can be expressed as:

(6) $$\begin{array}{c} S\left(r_{k}\right)=\underset{r_{k}\neq r_{i}}{\sum }w\left(r_{i}\right)D_{r}\left(r_{k},r_{i}\right)\text{.} \end{array}$$

In the bee colony algorithm, after the bee leads the bee back to the information sharing area, according to the shared food source information, the following probability is calculated according to the following formula:

(7) $$\begin{array}{c} B_{D}=\left|\log\left(\frac{I_{b}}{I_{f}}\right)\right|+D_{FB}\text{.} \end{array}$$

That is to say, the higher the rate of return of honey source found by bees, the easier it is to be selected. In load balancing problem, the objective function should take the minimum value, that is, the lowest load corresponds to the higher rate of return, so the probability that ant *m* is followed on node *V* is:

(8) $$\begin{array}{c} \sigma =\sqrt{\ln\;\left(1+\frac{v_{r}}{m^{2}}\right)}\text{.} \end{array}$$

Follow the ants to select the leading ants to follow according to the following follow-up probability, and generate a new food source around the food source *m* as follows, and use the greedy selection method to determine the food source to be retained; that is, always select the higher yield.

(9) $$\begin{array}{c} \mu =\ln\left(\frac{m^{2}}{\sqrt{v_{r}+m^{2}}}\right)\text{.} \end{array}$$

To solve the problem of load balancing, the larger the node load, the less resources available for the representative node, and the slower the processing speed. Therefore, the pheromone increment of the *K* ant should be expressed as follows:

(10) $$\begin{array}{c} M_{k}=c_{k}^{d}M_{k-1}\text{.} \end{array}$$

After a week of cycling, update the pheromone:

(11) $$\begin{array}{c} T_{r}=\frac{1}{N}\overset{k}{\underset{i=i_{0}}{\sum }}r_{i}r_{i}^{T}\text{.} \end{array}$$

Taking the place of the mean as the starting point, the function value tends to gradually decrease from the middle to the left and right sides. Its function expression is as follows:

(12) $$\begin{array}{c} PR\left(k\right)=T_{r}\left(k\right)-V_{r}\left(k\right)\text{.} \end{array}$$

Hadoop uses Java open source to implement Google's GFS and Map Reduce. Because of its scalability and high fault tolerance, it is favored by industry and university research institutes. Many organizations use the Hadoop platform as their big data and cloud. The base platform for computing. The execution model also creates a computational barrier in the process that allows us to ensure that tasks are synchronized between producers and consumers when necessary. With the development of the times, the amount of data generated by people is constantly increasing. Running only some uncoupled tasks on independent computers has long been unable to meet people's requirements for data processing. In order to improve the utilization of idle computing resources, for computing resources that have been allocated to a certain queue, if the computing resources are still in an idle state, other queues can share the free resources fairly. Before the Hadoop cluster performs its tasks or new machines join the cluster, the performance of the nodes is evaluated by the DHP algorithm, combined with the hardware conditions of the nodes, and the proportion of data stored by each machine is obtained. If there is an idle task tracker in the system, it will judge the degree of hunger of each queue and give priority to the task with the lowest ratio. The computing capacity scheduling algorithm requires a very strict number of users. If the number of users is not limited, there will be a serious unfair situation of user resources. Load imbalance will lead to low overall cluster throughput, underutilization of resources, low resource utilization, and other issues. On the other hand, some requests submitted by the users can not be executed as soon as possible, which increases the response time.

## 5. Conclusions

This paper mainly studies the load balancing problem of Hadoop, an open-source cloud platform. Considering that in the process of job scheduling, the cluster load should be balanced in advance rather than related to when the load is seriously unbalanced, the task scheduling process in the Hadoop cluster is analyzed in detail. Aiming at the shortcomings of the fair scheduling algorithm, two improved ideas, delay waiting and machine learning, are proposed to improve the resource utilization and overall performance of the Hadoop platform. When assigning tasks to Reduce after the Map task is completed, it is necessary to assign tasks according to the performance of the nodes where Reduce is located. Experiments verify the effectiveness of the algorithm. The LBNP algorithm has greatly improved the efficiency of Reduce task execution and Job execution. The delay capacity scheduling algorithm ensures that most tasks reach localized scheduling, improves resource utilization, improves load balancing, and speeds up job completion time. For high-load nodes, tasks are not assigned, and when the next idle node comes, the nodes are evaluated until the tasks are all completed. At the same time, the update mechanism of pheromone is improved and dynamic regulation factors are added to the volatilization mechanism, so that the pheromone is adaptively updated according to the load of the cluster, and the iteration time is shortened while avoiding local optimization. In view of the fact that Hadoop's default partitioning strategy uses the Hash algorithm to divide data, this strategy shows obvious limitations in mediating load balancing for the uneven distribution of data density.

## Figures and Tables

**Figure 1:** Hadoop map reduce calculation model.

**Figure 2:** Average response time of each node in a single test.

**Figure 3:** REST-map reduce framework architecture.

**Figure 4:** Evaluation model.

**Figure 5:** Map reduce calculation process.

**Figure 6:** Individual fitness probability and selected random number.

**Figure 7:** Node load evaluation.

## Data Availability

The data underlying the results presented in the study are available within the manuscript.

## References

[1] Alanazi R., Alhazmi F., Chung H., Nah Y. (2020). A multi-optimization technique for improvement of Hadoop performance with a dynamic job execution method based on artificial neural network. *SN Computer Science*.

[2] Kalia K., Gupta N. (2021). Analysis of hadoop MapReduce scheduling in heterogeneous environment. *Ain Shams Engineering Journal*.

[3] Jiang Y., Huang Z., Tsang D. H. K. (2020). On power-peak-aware scheduling for large-scale shared clusters. *IEEE Transactions on Big Data*.

[4] Yao Y., Wang J., Sheng B. (2015). Self-adjusting slot configurations for homogeneous and heterogeneous hadoop clusters. *IEEE Transactions on Cloud Computing*.

[5] Xiong R., Luo J., Dong F. (2015). Optimizing data placement in heterogeneous Hadoop clusters. *Cluster Computing*.

[6] Tang Z., Du L., Zhang X., Yang L., Li K. (2021). AEML: an acceleration engine for multi-GPU load-balancing in distributed heterogeneous environment. *IEEE Transactions on Computers*.

[7] Rallapalli S., Gondkar R. R., Ketavarapu U. P. K. (2016). Impact of processing and analyzing healthcare big data on cloud computing environment by implementing hadoop cluster. *Procedia Computer Science*.

[8] Qureshi B., Javed Y., Koubaa A., Sriti M. F., Alajlan M. (2016). Performance of a low cost hadoop cluster for image analysis in cloud robotics environment. *Procedia Computer Science*.

[9] Xun Y., Zhang J., Qin X., Zhao X. (2017). FiDoop-DP: data partitioning in frequent itemset mining on hadoop clusters. *IEEE Transactions on Parallel and Distributed Systems*.

[10] Chen Y., Zhou Y., Taneja S., Qin X., Huang J. (2017). aHDFS: an erasure-coded data archival system for hadoop clusters. *IEEE Transactions on Parallel and Distributed Systems*.

[11] Hodor P., Chawla A., Clark A., Neal L. (2016). cl-dash: rapid configuration and deployment of Hadoop clusters for bioinformatics research in the cloud. *Bioinformatics*.

[12] Banu A., Yakub M. (2020). Evolution of big data and tools for big data analytics. *Journal of Interdisciplinary Cycle Research*.

[13] Qureshi N. M. F., Shin D. R., Siddiqui I. F., Chowdhry B. S. (2017). Storage-tag-Aware scheduler for hadoop cluster. *IEEE Access*.

[14] Javanmardi A. K., Yaghoubyan S. H., Bagherifard K., Nejatian S., Parvin H. (2021). A unit-based, cost-efficient scheduler for heterogeneous Hadoop systems. *The Journal of Supercomputing*.

[15] Lim J. B., Ahn J. S., Lee K. W. (2016). Performance modeling and analysis of a hadoop cluster for efficient big data processing. *Advanced Science Letters*.

[16] Strutz M., Heßling H., Streit A. (2017). Transforming a local medical image analysis for running on a hadoop cluster. *Procedia Computer Science*.

[17] Zhou Q., Wu D., Tang C., Rong C. (2014). STSHC: secure and trusted scheme for Hadoop cluster. *International Journal of High Performance Systems Architecture*.

[18] Zhang Y., Yao Y. X., Yang J. (2014). Build a fully distributed hadoop cluster based on VM scene. *Advanced Materials Research*.

[19] Singh R., Kaur P. J. (2016). Analyzing performance of Apache Tez and MapReduce with hadoop multinode cluster on Amazon cloud. *Journal of Big Data*.

[20] Yao Y., Gao H., Wang J., Sheng B., Mi N. (2021). New scheduling algorithms for improving performance and resource utilization in hadoop YARN clusters. *IEEE Transactions on Cloud Computing*.

[21] Ibrahim S., Moise D., Chihoub H. E. (2014). Towards efficient power management in MapReduce: investigation of CPU-frequencies scaling on power efficiency in hadoop. *Lecture Notes in Computer Science*.

[22] Li Y., Tang B., Jiang X., Yi Y. (2022). Bearing fault feature extraction method based on GA-VMD and center frequency. *Mathematical Problems in Engineering*.

[23] Li Y., Mu L., Gao P. (2022). Particle swarm optimization fractional slope entropy: a new time series complexity indicator for bearing fault diagnosis. *Fractal Fract*.

[24] Bawankule K. L., Dewang R. K., Singh A. K. (2021). Historical data based approach for straggler avoidance in a heterogeneous Hadoop cluster. *Journal of Ambient Intelligence and Humanized Computing*.

[25] Bawankule K. L., Dewang R. K., Singh A. K. (2021). *Load Balancing Approach for a MapReduce Job Running on a Heterogeneous Hadoop Cluster, International Conference on Distributed Computing and Internet Technology*.

[26] Rani, R., Garg R., Singh A. K. (2021). A survey of thermal management in cloud data centre: techniques and open issues. *Personal Communications*.

[27] Hussein A. A. (2020). Using hadoop technology to overcome big data problems by choosing proposed cost-efficient scheduler algorithm for heterogeneous hadoop system (BD3). *Journal of Scientific Research and Reports*.

[28] Goswami A., Thakur D., Sharma P. Improving performance in hadoop cluster over cloud computing environment using hold & release mechanism.

[29] Dadheech P., Goyal D., Srivastava S., Kumar A. Performance improvement of heterogeneous hadoop clusters using query optimization.

[30] Chakravarthy N. S. K., Sudhakar N., Reddy E. S. (2018). An intelligent storage optimization technique for heterogeneous hadoop clusters. *International Journal of Simulation. Systems, Science and Technology*.

[31] Luo X., Fu X. (2019). Configuration optimization method of Hadoop system performance based on genetic simulated annealing algorithm. *Cluster Computing*.

[32] Padmanaban R., Mukesh R. (2020). Hadoopsec: sensitivity-aware secure data placement strategy for big data/hadoop platform using prescriptive analytics. *GSTF Journal on Computing*.

